# Effect of Systematic Holistic Nursing Combined with the MDT Teaching Method in the Nursing of Neonatal Jaundice and Its Impact on the Recovery of the Newborns' Physiological Function

**DOI:** 10.1155/2021/2013233

**Published:** 2021-12-10

**Authors:** Jie Dai, Yan Xu, Qigai Yin, Jing Chen, Haitang Shi, Yue Li

**Affiliations:** ^1^Nursing Unit of Department of Neonatology, The First People's Hospital of Lianyungang, The First Affiliated Hospital of Kangda College of Nanjing Medical University (The First People's Hospital of Lianyungang), Lianyungang 222000, Jiangsu Province, China; ^2^Nursing Department, The First People's Hospital of Lianyungang, The First Affiliated Hospital of Kangda College of Nanjing Medical University (The First People's Hospital of Lianyungang), Lianyungang 222000, Jiangsu Province, China; ^3^Department of Neonatology, The First People's Hospital of Lianyungang, Lianyungang 222000, Jiangsu Province, China; ^4^Pediatric Internal Medicine Nursing Unit, The First People's Hospital of Lianyungang, The First Affiliated Hospital of Kangda College of Nanjing Medical University (The First People's Hospital of Lianyungang), Lianyungang 222000, Jiangsu Province, China

## Abstract

The application effect of systematic holistic nursing combined with the multidisciplinary team (MDT) in the nursing of neonatal jaundice was explored. This study was a retrospective control study. 90 cases of neonatal jaundice admitted to our hospital (February 2020–February 2021) were equally split into group P treated with routine nursing and group Q treated with systematic holistic nursing combined with MDT. The application effect of the two nursing programs was compared and analyzed. Groups P and Q showed no statistical difference in general data (*P* > 0.05). Compared with group P, the jaundice regression time, hospitalization time, time of first defecation, and time of meconium turning yellow of group Q were notably shorter, and the body weight and total treatment efficiency of group Q were notably higher (*P* < 0.05). From the third day, the daily jaundice indexes between the two groups were different; that is, the indexes of group Q were notably lower compared with group P (*P* < 0.05). The scores of environmental nursing, special nursing, basic nursing, and service attitude in group Q were notably higher compared with group P (*P* < 0.05). In the nursing process of neonatal jaundice, the combination of systematic holistic nursing and MDT can effectively shorten the time of first defecation and meconium turning yellow, reduce jaundice indexes, promote the recovery of the physiological function, and improve the clinical efficacy and nursing quality.

## 1. Introduction

Neonatal jaundice is also known as hyperbilirubinemia, which is common in newborns at 2-3 days of age. It will cause the yellow staining of skin, sclera, and mucosa due to the abnormal bilirubin metabolism [1–3]. Mild jaundice may regress spontaneously. Pathological jaundice can damage the central nervous system of the newborns, easily lead to sequelae such as septicemia, hepatitis, and pneumonia, adversely affect their intelligence and motor function, and even endanger their life safety [4–7]. According to the current research status in this field, the exploration of therapeutic methods and nursing patterns of neonatal jaundice is still the research priority, and its main purpose is to ensure the improvement of the therapeutic outcome. Bowassa and other scholars [8] stated in their reports that systematic holistic nursing is very effective in the nursing process of neonatal jaundice. This paper believes that neonatal jaundice is a disease involving multiple disciplines such as neonatology, internal medicine, dermatology, nutrition, and psychology. If multidisciplinary team (MDT) nursing pattern can be established, it will be more conducive to strengthening cooperation between various disciplines, but currently, there are few reports about the application of MDT pattern in neonatal disease. Based on this, this study combined the MDT teaching method with systematic holistic nursing to explore its application effect in the nursing of neonatal jaundice. Under the MDT pattern, the nursing quality management system was tried to be constructed to truly achieve the comprehensive, whole-course, and high-quality nursing service. In order to further respond to the call of the National Medical Administration and Hospital Authority and enhance the development of nursing discipline in the nursing field of neonatal jaundice, this paper explored the application effect of systematic holistic nursing combined with MDT in nursing of neonatal jaundice. It aimed to adapt to the formation of the quality management system of multidisciplinary collaborative nursing under the new development phase and promote stable and orderly development of nursing in our country.

## 2. Materials and Methods

The inclusion criteria were as follows: ① the newborns who met clinical diagnostic criteria of pathological jaundice; ② the full-term newborns; ③ the newborns who met indications of blue light irradiation; ④ the breast-feeding newborns; ⑤ the newborns without abnormal liver function; ⑥ the family members of the newborns understood, agreed, and voluntarily participated in this study. The exclusion criteria were as follows: ① the newborns who had a history of asphyxia at birth; ② the newborns with congenital disease; ③ the newborns with serious and unstable condition; ④ the newborns with serious organic diseases. As we know, inclusion criteria mean that prospective participants must have if they want to join the study. The exclusion criteria mean that characteristics disqualify prospective participants from joining a study.

### 2.1. Screening and Grouping of Newborns

90 cases of neonatal jaundice admitted to our hospital (February 2020–February 2021) were selected and equally split into group P treated with routine nursing and group Q treated with systematic holistic nursing combined with MDT. The ethics committee of our hospital approved and supervised the implementation process of the study.

### 2.2. Methods

Group P was treated with routine nursing, that is, routine symptomatic and supportive treatment. The bilirubin levels of neonatal cord blood were regularly checked, and blue light therapy was conducted. The newborns' eyes and perineum were covered with a black cloth, and then the newborns were placed in a 420–480 nm phototherapy warmer and irradiated for 12 hours, with an interval of 12 hours. The changes of newborns' vital signs needed to be closely monitored.

Group Q was treated with systematic holistic nursing combined with the MDT teaching method, with the specific steps as follows. (1) Establishment of MDT teams: MDT teams [9–13] were made up of neonatal doctors, head nurses of the neonatal intensive care unit (NICU), pediatric nutritionists, psychologists, and five nursing staff in the neonatal department. (2) MDT nursing training: the training included the attention items of jaundice nursing, symptomatic nursing measures for related complications, the use of the Newborn Early Warning Score (NEWS) scale, concepts and methods of MDT nursing, communication with parents, and intervention techniques. The work plan of the MDT was clarified, the team meetings were held regularly, the effect evaluation and revision plan of treatment and nursing programs were timely conducted, problems were identified, and measures were improved [14–16]. (3) Routine nursing was strengthened based on the MDT concept. ① The levels of serum bilirubin, changes of vital signs, and the condition of skin, pupils, and the second defecation were closely monitored. The nursing measures such as phototherapy and hydrotherapy were improved. Nutrition plan was made with the help of pediatric nutritionists. The nursing process of skin, oral cavity, disinfection, and feeding was improved. Based on all of the above, NEWS scale was used to evaluate the disease condition of the newborns, which included body temperature, respiration, heart rate, consciousness, skin condition, and serum bilirubin level, with a total score of 15 points. Higher score indicated more serious condition. Zero points represented grade I monitoring, and routine NICU observation was performed, with observation and evaluation once every 2 h. 1-2 points represented grade II monitoring; that is, potential risks were prevented, related nursing was performed, and the frequency of dynamic assessment was increased, with once every hour. Three points and above represented grade III monitoring, and there was more intervention of doctors, team consultation, determination of treatment and nursing programs, and 24 h real-time monitoring. (4) Prevention and nursing of complications: ① the fluctuation degree of transcutaneous bilirubin and serum transaminase was monitored, and the stool color and defecation frequency were recorded in detail to prevent complications such as biliary atresia, neonatal pneumonia, septicemia, and hepatitis. ② Strict disinfection plan was performed to prevent cross-infection. (5) Reasonable emotional intervention for family members: it was completed with the help of psychologists and nursing staff. In the initial period of nursing, the psychologists communicated with the family members in detail, and the nursing staff made relevant records to gain insight into their understanding of neonatal jaundice and their current psychological state and comprehensively analyze the causes of their adverse emotions. According to the family members' actual condition, health education was carried out. They were informed of the newborns' disease condition and treatment programs, given spiritual support, guided to find out rational beliefs, and comforted by listing successful cases to avoid their overwhelming worry. Under the condition of disinfection, nursing and treatment instructions were made, and visitation was allowed to improve family support.

### 2.3. Observation Indexes

The gender, days of age, birth weight, disease severity, serum bilirubin level, intravenous infusion time, Apgar score and a number of natural childbirth, and age and education degree of maternal women were recorded. The basic clinical indicators including jaundice regression time, hospitalization time, and the changes of body weight of the newborns were recorded. The defecation condition including time of first defecation and meconium turning yellow of the newborns was analyzed.

If the neonatal jaundice disappeared, the time of meconium turning yellow was ≤3 h, and the serum bilirubin level was ≤119.7 *μ*mmol/L, it was markedly effective. If the neonatal jaundice basically disappeared, the time of meconium turning yellow was 3–5 h, and the serum bilirubin level was 119.7–171.0 *μ*mmol/L, it was effective. If the neonatal jaundice was not improved or aggravated, it was invalid. The total effective rate = (effective cases + markedly effective case)/the total cases × 100%.

The transcutaneous jaundice meter was used to detect the jaundice indexes of the two groups of newborns within 5 days. After nursing intervention, our self-made questionnaire on the nursing quality of neonatal jaundice was used to evaluate the nursing quality of the two nursing programs. The survey objects were family members of the newborns, and the survey content included environmental nursing, special nursing, basic nursing, and service attitude, with each part of 15 points. The score was proportional to the nursing quality. The preexperimental evaluation of the questionnaire had a consistency reliability of 0.91 and a validity coefficient of 0.80.

### 2.4. Statistical Treatment

In this study, SPSS 22.0 was used to calculate the differences between groups, and selected drawing software was GraphPad Prism 7 (GraphPad Software, San Diego, USA). This study included count data and measurement data. The count data were tested by *X*^2^ test and described by *n* (%). The measurement data were tested by *t*-test and described by ($\bar{x}$ ± *s*). *P* < 0.05 indicated that the difference had statistical significance.

## 3. Results

### 3.1. General Data

After statistical treatment, the comparison of general information between the two groups showed *P* > 0.05; that is, the difference was not significant, indicating comparability (see Table 1).

### 3.2. Basic Clinical Indicators

After nursing, compared with group P, the jaundice regression time and hospitalization time of group Q were notably shorter, but the body weight of group Q was notably higher (*P* < 0.05). The difference had statistical significance (see Table 2).

### 3.3. Defecation Condition

The time of first defecation and meconium turning yellow of group Q was notably shorter compared with group P (*P* < 0.05), and the difference had statistical significance (see Figure 1).

### 3.4. Clinical Efficacy

The total treatment efficiency in group Q was notably higher compared with group P (*P* < 0.05), and the difference had statistical significance (see Figure 2).

### 3.5. Jaundice Indexes

From the third day, the daily jaundice indexes between the two groups were different; that is, the indexes of group Q were notably lower compared with group P (*P* < 0.05) (see Figure 3).

### 3.6. Nursing Quality

The scores of environmental nursing, special nursing, basic nursing, and service attitude in group Q were notably higher compared with group P (*P* < 0.05). The difference had statistical significance (see Table 3).

## 4. Discussion

The treatment and rehabilitation of many diseases cannot be completed by a single discipline or major due to their complexity and the specialization of treatment technology, as well as the changes of diagnosis and treatment thoughts. Neonatal jaundice is a common neonatal disease, which is closely related to abnormal bilirubin metabolism, with many causes and extremely complex pathological types [17–20]. The severe pathological jaundice can cause systemic symptoms such as mental fatigue, poor response, anorexia, abnormal muscular tension, irritability, breathing difficulties, and convulsion, which is easy to damage the central nervous system and cause sequelae. Death can be caused in severe cases. Relevant studies have shown that nursing is an important method to promote the recovery of neonatal jaundice. Systematic holistic nursing has passed a number of clinical tests, which confirms its necessity in the nursing process of neonatal jaundice [21–24].

This study showed that, compared with group P, the jaundice regression time, hospitalization time, time of first defecation, and time of meconium turning yellow of group Q were notably shorter, and the body weight of group Q was notably higher (*P* < 0.05). It indicated that the combination of systematic holistic nursing and MDT could effectively improve the defecation condition and promote the jaundice regression. Systematic holistic nursing pays much attention to the changes of vital signs, rate of disease progression, location of jaundice, range, disease severity, and color of defecation and formulates complete individualized preconditioning measures according to common clinical manifestations. Under the guidance of MDT, the degree of neonatal nutrition intervention was improved, the newborns' food intake was appropriately increased according to their actual condition, and excretion of conjugated bilirubin was accelerated by promoting discharge of meconium, which were the main reasons why the body weight of group Q increased after nursing. In addition, the total treatment efficiency of group Q was notably higher compared with group P (*P* < 0.05), which tallied with the research of Kane and Luz [25]. From the third day, the daily jaundice indexes between the two groups were different; that is, the indexes of group Q were notably lower compared with group P (*P* < 0.05). The scores of environmental nursing, special nursing, basic nursing, and service attitude in group Q were notably higher compared with group P (*P* < 0.05). Analysis of the reasons is as follows: ① during the treatment, nursing staff closely observed the newborns' physical signs, frequently communicated with neonatal doctors, and supplied trace elements to keep water and electrolyte balance. During nursing, microbial ecological agent, phenobarbital, etc., was used to promote bile excretion to balance body's microflora. It reflected the collaboration between paediatrics and internal medicine under the guidance of MDT, which further guaranteed the therapeutic effect in the nursing process. ② During the treatment, nursing staff provided auditory and tactile comfort to newborns under the guidance of psychologists to improve their treatment compliance. At the same time, the psychologists carried out effective psychological intervention for maternal women and their family members, which increased their awareness of jaundice, improved their cooperation, and increased external support for therapy. It reflected the collaboration between nursing and psychology under the guidance of the MDT. Thus, it can be seen that the combination of systematic holistic nursing and MDT can effectively improve the therapeutic effect of neonatal jaundice.

## 5. Conclusion

In the nursing process of neonatal jaundice, the combination of systematic holistic nursing and MDT can effectively shorten the time of first defecation and meconium turning yellow, reduce jaundice indexes, promote the recovery of the physiological function, and improve the clinical efficacy and nursing quality.

However, this study still has some limitations. ① This study was a retrospective analysis study. After hospital discharge, for most newborns, the follow-up time was short, and continuous nursing was not available. ② The sample size selected in this paper was small due to research cost, so it is necessary to expand the sample to carry out multicenter research in the future.

## Figures and Tables

**Figure 1:** Comparison of defecation condition between group P and group Q (*n* = 45, $\bar{x}$ ± *s*). *Note.* The horizontal axis represented evaluation dimension, namely, the time of first defecation and time of meconium turning yellow, and the vertical axis represented time (h). The time of first defecation and meconium turning yellow of group P was 17.81 ± 3.60 and 56.91 ± 6.21, respectively. The time of first defecation and meconium turning yellow of group Q was 6.25 ± 1.85 and 30.01 ± 2.54, respectively. *∗* indicated that there was a significant difference in the time of first defecation between the two groups (*t* = 19.1591, *P* < 0.001). *∗∗* indicated that there was a significant difference in the time of meconium turning yellow between the two groups (*t* = 26.8953, *P* < 0.001).

**Figure 2:** Analysis of clinical efficacy between group P and group Q (*n* (%)). *Note.* In group P, 10 cases were invalid, 19 were effective, and 16 were markedly effective, with the total effective cases of 35. In group Q, 2 cases were invalid, 18 were effective, and 25 were markedly effective, with the total effective cases of 43. ∗ indicated that there was an obvious difference in the total treatment efficiency between the two groups (*X*^2^ = 6.1538, *P*=0.013).

**Figure 3:** Analysis of jaundice indexes between group P and group Q (*n* = 45, $\bar{x}$ ± *s*). *Note.* The horizontal axis represented time nodes, and the vertical axis represented jaundice indexes (ml/dI). In group P, the jaundice indexes from day 1 to 5 were 6.37 ± 1.03, 7.34 ± 1.26, 9.29 ± 1.78, 12.76 ± 1.42, and 13.91 ± 2.45, respectively. In group Q, the jaundice indexes from day 1 to 5 were 6.42 ± 1.02, 7.28 ± 1.35, 8.11 ± 1.20, 9.22 ± 1.34, and 9.08 ± 1.27, respectively. *∗* from left to right indicated that the jaundice indexes of the two groups on the 3rd, 4th, and 5th day were significantly different (*t* = 3.6873, 12.1628, and 11.7411; all showed *P* < 0.05).

**Table 1:** Comparison of general data (*n* = 45).

Items	Group P	Group Q	*X* ^2^/*t*	*P*
Gender (boy/girl)	20/25	22/23	0.1786	0.673
Days of age (d)	5.51 ± 0.51	5.49 ± 0.48	0.1916	0.8485
Birth weight (kg)	3.31 ± 0.21	3.26 ± 0.18	1.2127	0.2285
Disease severity				
Mild degree	13 (28.89)	12 (26.66)	0.0554	0.814
Moderate degree	25 (55.56)	24 (53.33)	0.0448	0.832
Severe degree	7 (15.56)	9 (20)	0.3041	0.581
Bilirubin levels (*μ*mmol/L)	247.84 ± 14.37	251.02 ± 15.13	1.0223	0.3094
Jaundice indexes (mg/dI)	22.38 ± 1.05	22.47 ± 1.19	0.3804	0.7045
Number of natural childbirth	24 (53.33)	22 (48.89)	0.1779	0.673
Intravenous infusion time (d)	5.59 ± 2.41	5.62 ± 2.51	0.0578	0.9540
Apgar scores	8.34 ± 1.05	8.42 ± 1.03	0.3649	0.7161
Age of maternal women (years)	32.44 ± 5.02	30.86 ± 5.17	1.4708	0.1449
Education degree of maternal women				
Below junior middle school	6 (13.33)	3 (6.67)	1.1111	0.292
Junior middle school to senior high school	21 (46.67)	20 (44.44)	0.0448	0.832
Above senior high school	18 (40)	22 (48.89)	0.7200	0.396

**Table 2:** Analysis of basic clinical indexes (*n* = 45, $\bar{x}$ ± *s*).

Items	Jaundice regression time (d)	Hospitalization time (d)	Body weight (kg)
Group P	8.74 ± 2.06	10.01 ± 2.04	3.25 ± 0.26
Group Q	5.62 ± 1.35	6.13 ± 1.47	3.50 ± 0.22
*t*	8.4978	10.3513	4.9240
*P*	<0.001	<0.001	<0.001

**Table 3:** Analysis of nursing quality (*n* = 45, $\bar{x}$ ± *s*).

Items	Environmental nursing	Special nursing	Basic nursing	Service attitude
Group P	10.14 ± 1.45	9.32 ± 1.51	10.63 ± 2.11	8.44 ± 2.23
Group Q	13.47 ± 1.09	11.61 ± 1.35	13.06 ± 1.76	13.05 ± 1.62
*X* ^2^/*t*	12.3144	7.5842	5.9326	11.2196
*P*	<0.001	<0.001	<0.001	<0.001

## Data Availability

The datasets used and/or analyzed during the current study are available from the corresponding author upon reasonable request.

## References

[1] Blythe J. (2018). Short report-the MDT speed date. *Creative Education*.

[2] Magee L., Roberts J., Beattie V., De Normanville C., Borthwick D. (2016). 97 Using Your Voice 2014 - how to use your nursing voice at the MDT. *Lung Cancer*.

[3] Peterson J., Jung J., Hoffman L., David R. (2016). Nursing management of maggot debridement therapy (MDT) for wound debridement in patients with chronic graft versus host disease wounds. *Biology of Blood and Marrow Transplantation*.

[4] Dantas A. V. V. C., Farias L. J. R., de Paula S. J. (2018). Nursing diagnosis of neonatal jaundice: study of clinical indicators. *Journal of Pediatric Nursing*.

[5] Selalmaz M., Bulbul A., Sozeri S. (2015). The evaluation of the implementation level of nurses working in neonatal intensive care unit in the treatment of neonatal jaundice. *Şişli Etfal Hastanesi Tip Bülteni*.

[6] Gundur N. M., Kumar P., Sundaram V., Thapa B. R., Narang A. (2010). Natural history and predictive risk factors of prolonged unconjugated jaundice in the newborn. *Pediatrics International*.

[7] Maisels M. J., Coffey M. P., Gendelman B. (2016). Diagnosing jaundice by eye-outpatient Assessment of conjunctival icterus in the newborn. *The Journal of Pediatrics*.

[8] Bowassa G. E., Ngono G. T. W., Ngakengni N. Y. (2019). Jaundice in the newborn at the teaching hospital of brazzaville. *Open Journal of Pediatrics*.

[9] Aydin D., Karaca Ciftci E., Karatas H. (2014). Identification of the traditional methods of newborn mothers regarding jaundice in Turkey. *Journal of Clinical Nursing*.

[10] Carvalho O. M. C., Augusto M. C. C., Medeiros M. Q. (2019). Late umbilical cord clamping does not increase rates of jaundice and the need for phototherapy in pregnancies at normal risk. *Journal of Maternal-Fetal and Neonatal Medicine*.

[11] Bice A. A., Wyatt T. H. (2017). Holistic comfort interventions for pediatric nursing procedures: a systematic review. *Journal of Holistic Nursing*.

[12] Lange B., Zahourek R. P., Mariano C. (2014). A legacy building model for holistic nursing. *Journal of Holistic Nursing*.

[13] Papadopoulou C., Sime C., Rooney K., Kotronoulas G. (2019). Sexual health care provision in cancer nursing care: a systematic review on the state of evidence and deriving international competencies chart for cancer nurses. *International Journal of Nursing Studies*.

[14] Zahed Pasha Y., Alizadeh-Tabari S., Zahed Pasha E., Zamani M. (2020). Etiology and therapeutic management of neonatal jaundice in Iran: a systematic review and meta-analysis. *World Journal of Pediatrics*.

[15] Senyüz O. F., Yeşildağ E., Emir H. (2001). Diagnostic laparoscopy in prolonged jaundice. *Journal of Pediatric Surgery*.

[16] Wagh V. V., Jain A. K. (2016). *Ethnomedicine for Curing Jaundice in Jhabua District of MadhyaPradesh*.

[17] Fan Y., Wu S. D., Kong J. (2013). Obstructive jaundice and melena caused by hemocholecyst: a case report. *World Journal of Gastroenterology*.

[18] Nussenzveig R. H., Christensen R. D., Prchal J. T., Yaish H. M., Agarwal A. M. (2014). Novel *α*-smt causing severe neonatal jaundice from hereditary spherocytosis. *Neonatology*.

[19] Trutin I., Valent Morić B., Borošak J., Stipančić G. (2018). Does urinary tract ultrasound have its place in the treatment of early neonatal jaundice? Neonatal bilateral adrenal hemorrhage: case report. *Acta Clinica Croatica*.

[20] Gupta R., Anand A., Kumar M., Bhatt M., Singh S., Sonkar A. A. (2018). Safety and efficacy of low-dose single-agent capecitabine in inoperable gallbladder cancer with jaundice post-single-system single-catheter external biliary drainage: a pilot study from a highly endemic area. *Indian Journal of Surgical Oncology*.

[21] Pan X., Li L., Lin H. (2019). A graphene oxide-gold nanostar hybrid based-paper biosensor for label-free SERS detection of serum bilirubin for diagnosis of jaundice. *Biosensors and Bioelectronics*.

[22] Lowes M., Kleiss M., Lueck R. (2017). The utilization of multidisciplinary tumor boards (MDT) in clinical routine: results of a health care research study focusing on patients with metastasized colorectal cancer. *International Journal of Colorectal Disease*.

[23] Epstein J. (2013). The calculus concept inventory-measurement of the effect of teaching methodology in mathematics. *Notices of the American Mathematical Society*.

[24] Malhotra P., Lovell N., Plant P. K., Callister M. E. J., Karthik S., Scarsbrook A. (2011). P162 Comparison of clinical characteristics and outcomes of patients with PET positive vs PET negative solitary pulmonary nodules managed by a Lung MDT. *Australian and New Zealand Journal of Psychiatry*.

[25] Kane B., Luz S. (2013). “Do no harm”: f. *International Journal of Medical Informatics*.

